# Fibroblast growth factors 7 and 10 are involved in ameloblastoma proliferation via the mitogen-activated protein kinase pathway

**DOI:** 10.3892/ijo.2013.2081

**Published:** 2013-08-29

**Authors:** YU NAKAO, TAKESHI MITSUYASU, SHINTARO KAWANO, NORIFUMI NAKAMURA, SHIORI KANDA, SEIJI NAKAMURA

**Affiliations:** 1 Section of Oral and Maxillofacial Oncology, Division of Maxillofacial Diagnostic and Surgical Sciences, Faculty of Dental Science, Kyushu University, Fukuoka;; 2 Department of Oral and Maxillofacial Surgery, Graduate School of Medical and Dental Sciences, Kagoshima University, Kagoshima, Japan

**Keywords:** ameloblastoma, tooth development, fibroblast growth factor, AM-1, MAPK pathway

## Abstract

Ameloblastoma is an epithelial benign tumor of the odontogenic apparatus and its growth mechanisms are not well understood. Fibroblast growth factor (FGF) 3, FGF7 and FGF10, which are expressed by the neural crest-derived ectomesenchymal cells, induce the proliferation of odontogenic epithelial cells during tooth development. Therefore, we examined the expression and function of these FGFs in ameloblastoma. We examined 32 cases of ameloblastoma as well as AM-1 cells (an ameloblastoma cell line) and studied the expression of FGF3, FGF7, FGF10 and their specific receptors, namely, FGF receptor (FGFR) 1 and FGFR2. Proliferation, mitogen-activated protein kinase (MAPK) signaling and PI3K signaling were examined in AM-1 cells after the addition of FGF7, FGF10 and these neutralizing antibodies. The expression of FGF7, FGF10, FGFR1 and FGFR2 was detected in ameloblastoma cells and AM-1 cells, while that of FGF3 was not. FGF7 and FGF10 stimulated AM-1 cell proliferation and phosphorylation of p44/42 MAPK. However, Akt was not phosphorylated. Blocking the p44/42 MAPK pathway by using a specific mitogen-activated protein/extracellular signal-regulated kinase (MEK) inhibitor (U0126) completely neutralized the effects of FGF7 and FGF10 on AM-1 cell proliferation. However, Anti FGF7 and FGF10 neutralizing antibodies did not decrease cell proliferation and MAPK phosphorylation of AM-1 cells. These results suggested that FGF7 and FGF10 are involved in the proliferation of ameloblastoma cells through the MAPK pathway.

## Introduction

Ameloblastoma is a benign tumor of the jaw that is characterized by local invasion and a high tendency to recur. This tumor is thought to arise from the odontogenic epithelial apparatus or its remnant tissues and has a histological appearance similar to the developing enamel organ (1–3). However, in spite of numerous histological and biological studies, the mechanisms underlying the proliferation of this tumor are still poorly understood.

Fibroblast growth factors (FGFs) have important proliferative functions in the development of limbs, lungs, hair and feathers, as well as in wound healing and development of some tumors (4–10). In mammals, the FGF family currently consists of 23 structurally related growth factors (11), the biological effects of which are mediated through 4 high-affinity tyrosine kinase receptors, called fibroblast growth factor receptors (FGFR) 1–4. FGFR1-3 have RNA isoforms produced through alternative splicing and have different ligand-binding properties (12–14). In the developing tooth germ, the proliferation and differentiation are governed by interactions between the odontogenic epithelium and the neural crest-derived ectomesenchyme including the FGF signaling (15–18). Among the FGFs, FGF3, FGF7 and FGF10 are expressed in mesenchymal cells and have important roles in the proliferation of odontogenic epithelial cells during tooth development (19–21). FGF3 stimulates the proliferation of inner enamel epithelial cells, FGF7 also stimulates the proliferation of outer enamel epithelial cells and FGF10 maintains dental epithelial stem cells (22,23). FGF7 binds to FGFR2 only, while FGF3 and FGF10 bind to both FGFR1 and FGFR2 (24,25). Signaling through FGFR1 and FGFR2 causes activation of the mitogen-activated protein kinases (MAPKs) and phosphoinositide 3-kinase (PI3K). When FGF binds its receptors, MAPK are stimulated to phosphorylate Raf, MEK and ERK sequentially. Finally, activated ERK translocates to the nucleus, activates transcription factors and induces cell proliferation. PI3K is also phosphorylated downstream of FGF, resulting in the phosphorylation of Akt and the inhibition of apoptosis (26).

In the present study, we thus hypothesized that FGF3, FGF7 and FGF10 may also affect the proliferation of ameloblastoma cells with odontogenic epithelial characteristics and show some evidences that FGF signaling involved in the ameloblastoma proliferation through MAPK pathway.

## Materials and methods

### Tissue samples and AM-1 cell culture

Surgically resected ameloblastoma tissues, with written consent, from 32 patients (20 men and 12 women), from the mandibles (31 cases) and maxilla (1 case), were analysed. Tissue samples were classified according to the World Health Organization’s International Histological Typing of Odontogenic Tumors, 2nd edition: 18 cases, follicular type; 8 cases, plexiform type; 4 cases, basal cell type; and 2 cases, desmoplastic type. Resected samples were fixed in a 4% paraformaldehyde (PFA) solution for 24–48 h and embedded in paraffin. To prepare frozen samples, tissues were embedded in OCT compound (Tissue-Tek; Sakura Finetechnical Co., Tokyo, Japan), frozen in liquid nitrogen and stored at −80°C. Paraffin sections were sliced at 4-*μ*m thickness and the frozen sections were sliced at 6-*μ*m thickness; sections were then mounted on poly-L-lysine-coated glass slides for immunohistochemical studies. AM-1 cells, an immortalized ameloblastoma cell line transfected with HPV-16 DNA, were used in this study (27). They were cultured in Keratinocyte-SFM medium (Gibco Invitrogen Corp., Carlsbad, CA, USA), which were calcium chloride free medium for inhibiting cell differentiation, containing 1% penicillin-streptomycin (Gibco), 0.2% fungizone amphotericin B (Gibco) and bovine pituitary extract (Gibco BRL, Grand Island, NY, USA) at 37°C in a humidified atmosphere containing 5% CO_2_.

### Immunohistochemistry

Paraffin-embedded tissue sections were de-paraffinized, frozen sections were fixed in 4% PFA for 30 min and AM-1 cells cultured on Lab-Tek Chamber Slides (Nalge Nunc International, Naperville, IL, USA) and fixed with acetone: 99.5% ethanol (1:1) for 15 min. Slides were then immersed in 3% hydrogen peroxide for 30 min and 10% normal goat serum prepared in phosphate-buffered saline (PBS) for 20 min. The primary antibodies (Table I) were applied overnight in a moist chamber at 4°C, labeled using a Histofine SAB-PO (R) kit (Nichirei Co., Tokyo, Japan) and visualized with diaminobenzidine (Nichirei). Negative controls were prepared by substituting PBS for primary antibody. Tissue sections were counterstained with hematoxylin. In each step, the samples were washed thrice with PBS for 5 min. According to their immunoreactivity, these samples were further classified into 3 groups; negative (−), weakly positive (+) and strongly positive (++).

### Reverse transcription-polymerase chain reaction (RT-PCR)

Total RNA was isolated from 10 cases of ameloblastoma (follicular type, 7; plexiform type, 1; basal cell type, 2) and AM-1 cells by using a QuickPrep Total RNA Extraction kit (Amersham Biosciences, Piscataway, NJ, USA). mRNA was transcribed to cDNA by using Ready-to-go You-Prime First-Strand Beads (Amersham Biosciences) and random primers, according to the manufacturer’s instructions. Primer sequences are listed in Table II. PCR was performed using Ready-To-Go PCR beads. Diethylpyrocarbonate water (26 *μ*l), forward primer (1 *μ*l) and reverse primer (1 *μ*l) were added to the beads. PCR of FGF3, FGF7 and β-actin was carried out for 30 cycles at 95°C for 30 sec, 55°C for 1 min and 72°C for 1 min, while that of FGF10 was carried out for 30 cycles at 95°C for 45 sec, 65°C for 45 sec and 72°C for 45 sec. The PCR products were separated on 2% agarose gels and stained with ethidium bromide.

### Immunoblotting

Fresh tissue samples from 4 cases (follicular type, 2; plexiform type, 1; basal cell type, 1) of ameloblastoma and AM-1 cells were homogenized and lysed in a buffer containing 20 mM HEPES/NaOH (pH 7.2), 150 mM NaCl, 2 mM EDTA, 1% Triton X-100, 50 mM sodium fluoride, 2 mM sodium orthovanadate, 30 mM sodium pyrophosphate and a mixture of protease inhibitors (10 *μ*M aprotinin, 10 *μ*M pepstatin A, 10 *μ*M leupeptin and 1 mM PMSF). For phosphorylation assays, AM-1 cells were seeded in Keratinocyte-SFM with pituitary extract for 24 h, washed with PBS and then incubated in Keratinocyte-SFM without bovine pituitary extract for 24 h, before being stimulated with recombinant FGF7 (Peprotech Inc., Rocky Hill, NJ, USA) or recombinant FGF10 (R&D Systems, Inc., Minneapolis, MN, USA) for the indicated time periods. In some experiments, cells were pre-incubated for 1 h with 1 or 10 *μ*M U0126 (a specific inhibitor of MEK1/2) (Cell Signaling Technology, Danvers, MA, USA). U0126 was dissolved in dimethyl sulfoxide (DMSO) and a similar concentration (0.1%) was added to PBS as a control, before treatment with the growth factor. The proteins were separated on a sodium dodecyl sulfate (SDS)-polyacrylamide gel and transferred to a nitrocellulose membrane. After the blocking of non-specific binding with 0.1% BSA in PBS, the membrane was incubated with the primary antibodies (Table I). Secondary antibodies were horseradish peroxidase-conjugated donkey anti-rabbit IgG antibodies (Amersham Biosciences) diluted 1:1,000 or donkey anti-mouse IgG antibody (Amersham Biosciences) diluted 1:2,000. The bound antibodies were visualized using the ECL system (Amersham Biosciences).

### Cell proliferation assay

AM-1 cells (2,500/well) were seeded in 96-well plates and then incubated in Keratinocyte-SFM with pituitary extract for 24 h. Cells were treated with FGF7 or FGF10, FGF7 (Abcam, Cambridge, UK) or FGF10 (Peprotech Inc.) neutralizing antibody and MAPK inhibitor (U0126) were added to the culture medium every 48 h. After treatment, the cells were enumerated using a Cell-Counting kit (Dojindo, Tokyo, Japan) according to the manufacturer’s instructions. Briefly, 10 *μ*l of the reagent was added to each well and incubated for 2 h. The reaction was measured at 450 nm by using a microplate reader.

### Statistical analyses

Results of proliferation assay were expressed as mean ± standard error of mean (SE). Data were analyzed by unpaired Student’s t-test. Statistical significance was set as p<0.05. Analyses were applied to experiments carried out at least three times.

## Results

### Expression of FGF7 and FGF10 in various types of ameloblastoma and AM-1 cells

*FGF7* and *FGF10* were expressed in all types of ameloblastoma and AM-1 cells, though expression of *FGF3* was not found (Fig. 1A). By western blot analyses, FGF7 and FGF10 were also detected in the ameloblastoma tissues and AM-1 cells (Fig. 1B). Furthermore, immunohistochemical location of FGF7 and FGF10 was investigated mainly in the stromal cells rather than the tumor cells (Fig. 1C and Table III).

### Localization of FGFR1 and FGFR2 in various types of ameloblastoma and AM-1 cells

Next, we performed immunohistochemistry to analyze the expression of FGFR1 and FGFR2, the specific receptors of FGF7 and FGF10, in the ameloblastoma specimens and in AM-1 cells. FGFR1 was expressed in the tumor and stromal cells of ameloblastoma, the expression of FGFR2 was investigated only in the tumor cells (Fig. 2). In the follicular ameloblastoma, FGFR1 was strongly expressed in the stromal cells (Table III). In AM-1 cells, the expression of FGFR1 and FGFR2 was detected in the cytoplasm and cell membrane (Fig. 2D and H). FGFR1 and FGFR2 were weakly expressed in the desmoplastic type tissues (Table III).

### Effect of recombinant human FGF7 and FGF10 proteins on cell proliferation and phosphorylation of p44/42 MAPK in AM-1 cells

When various concentrations (0, 1, 10 and 100 ng/ml) of recombinant human FGF7 or FGF10 proteins were added to the medium, AM-1 cells proliferated in a dose-dependent manner. At the highest dose of FGF7 and FGF10 (100 ng/ml), the number of cells increased to 176 and 247% of the control value, respectively (Fig. 3). The time course of p44/42 phosphorylation in AM-1 cells during treatment with FGF7 (10 ng/ml) and FGF10 (10 ng/ml) was examined using an anti-phospho-p44/42 MAPK antibody. FGF7-mediated activation of phospho-p44/42 MAPK peaked at 5 min and continued for up to 15 min (Fig. 4A). FGF10 caused increased p44/42 phosphorylation at 5 min that lasted for up to 30 min (Fig. 4B). Pre-treatment with the MAPK inhibitor U0126 completely inhibited the phosphorylation of p44/42 MAPK by FGF7 and FGF10 (Fig. 4C). Interestingly, phosphorylation of Akt (Ser473) through PI3K/Akt signaling pathway was not investigated by adding FGF7 or FGF10 (Fig. 4D). U0126 also inhibited proliferation of AM-1 cells stimulated with FGF7 or FGF10 (Fig. 5). Furthermore, to examine whether FGF7 and FGF10 secreted by AM-1 cells affect the proliferation through autocrine stimulation, neutralized antibodies for these FGFs were added to the culture of AM-1 cells. The addition of FGF7 or FGF10 neutralizing antibody did not inhibit the proliferation of AM-1 cells and the activation of phospho-p44/42 MAPK was not investigated (Fig. 6).

## Discussion

The expression of FGF1, FGF2, FGFR2 and FGFR3 in ameloblastoma was previously reported and it was concluded that FGF1 and FGF2 may contribute to the growth and development of ameloblastoma mediated by their receptors (27–29). However, the function of FGF signaling in ameloblastoma is still poorly understood, because these previous reports investigated only the expression patterns in this tumor immunohistochemically. In this study, we examined the expression of FGF3, FGF7, FGF10 and their specific receptors in histologically various types of ameloblastoma and analyzed the effect of these growth factors on the proliferation of ameloblastoma using the ameloblastoma cell line AM-1.

It is already known that FGF7 and FGF10 act as a proliferative signal from mesenchyme to epithelium through the FGFR1 and FGFR2 during tooth development (19). Immunohistochemical staining in the present study also revealed the expression of FGF7 and FGF10 mainly in the stromal cells rather than the tumor cells. Therefore, to examine the effects of FGF7 and FGF10 on the proliferation of ameloblastoma, cell proliferation assays were performed. The addition of recombinant human FGF7 or FGF10 proteins to the culture medium stimulated the proliferation of AM-1 cells in the dose-dependent manner. Our previous study also showed that FGF10 was expressed in the mesenchymal cells stimulating the proliferation of rat dental epithelial cells (21). Previously it was demonstrated that FGF10 induces cell migration and invasion in pancreatic cancer (30). Taken together, FGF7 and FGF10 may play important roles in the proliferation and progression of ameloblastoma.

In this study, the expression of FGF7 and FGF10 was also detected in AM-1 cells. To examine the effects of autocrine stimulation of FGF7 and FGF10 on the proliferation of AM-1, neutralized antibodies for these FGFs were thus added to the culture. However, adding FGF7 or FGF10 neutralizing antibody did not inhibit the proliferation of AM-1 cells. These results suggest that FGF7 and FGF10 may act as paracrine factors from stromal cells rather than autocrine factors from tumor cells in the proliferation of ameloblastoma.

MAPKs are evolutionarily conserved enzymes connecting cell-surface receptors to critical regulatory targets within the cells. In mammals, MAPK signaling cascades regulate important cellular processes. ERK1 (p/44) and ERK2 (p/42) are predominantly activated by mitogenic factors and they, in turn, activate transcription factors such as elk, c-myc and c-fos, which stimulate cell proliferation, differentiation and survival (31–34). In this study, we found that FGF7 and FGF10 induced the phosphorylation of p44/42 MAPK in AM-1 cells and U0126 inhibited this phosphorylation as well as the proliferation of AM-1 cells. On the other hand, phosphorylation of Akt was not confirmed. These results suggested that the MAPK pathway might have an important role in the FGF7- and FGF10-stimulated growth of ameloblastomas.

In conclusion, this study showed that FGF7 and FGF10 are expressed in ameloblastomas and that they play an important role in the growth of ameloblastomas through the MAPK pathway.

## Figures and Tables

**Figure 1.** Expression of FGF3, FGF7 and FGF10 in the ameloblastoma tissues and AM-1 cells. (A) RT-PCR method. FGF7 and FGF10 are expressed in the variety of ameloblastoma tissues and AM-1 cells, but FGF3 is not. (B) Western blot analysis. Expression of FGF7 and FGF10 is detected in the ameloblastoma and AM-1 cells. (C) Immunohistochemistry for FGF7 (a) and FGF10 (b) in the follicular type ameloblastoma. The intense expression FGF7 and FGF10 are investigated in the stromal cells rather than the tumor cells (×400).

**Figure 2.** Immunohistochemical location of FGFR1 and FGFR2 in the ameloblastoma specimens and AM-1 cells. Follicular type (A and E), plexiform type (B and F), basal cell type (C and G) and AM-1 cells (D and H) are shown (×200). FGFR1 is strongly expressed in the tumor cells of the plexiform type and stromal cells of the follicular and basal cell types (A–C), intense immunoreactivity for FGFR2 is detected only in the tumor cells (E–G). FGFR1 and FGFR2 are also expressed in AM-1 cells.

**Figure 3.** Effects of adding recombinant FGF7 and FGF10 proteins to the proliferating AM-1 cells. FGF7 (A) and FGF10 (B) stimulate the growth of AM-1 cells in a dose-dependent manner. AM-1 cells were treated with 0, 1, 10 or 100 ng/ml of FGF7 or FGF10 for 3 and 6 days. Results of the proliferation assay are expressed as mean ± SE. ^*^p<0.05, ^**^p<0.01.

**Figure 4.** Phosphorylation of p44/42 MAPK by the stimulation of FGF7 or FGF10 in AM-1 cells. AM-1 cells were stimulated with 10 ng/ml of FGF7 or FGF10 for 1, 5, 15, 30, 60 and 120 min. FGF7-mediated activation of phospho-p44/42 MAPK peaks at 5 min and continues for up to 15 min (A). FGF10 causes increased p44/42 phosphorylation at 5 min that lasts for up to 30 min (B). To inhibit the phosphorylation of p44/42 MAPK, 1 or 10 *μ*M U0126 was applied for 1 h before stimulation with 10 ng/ml of FGF7 or FGF10 for 5 min. Adding U0126 completely inhibited the phosphorylation of p44/42 MAPK by FGF7 and FGF10 stimulation (C). To examine Akt phosphorylation, AM-1 cells were stimulated with 10 ng/ml of FGF7 or FGF10. The phosphorylation of Akt was not investigated by the stimulation of FGF7 or FGF10 (D).

**Figure 5.** Inhibition of the FGF7 or FGF10-stimulated growth by MAPK inhibitor U0126 in AM-1 cells. AM-1 cells were treated with 1 or 10 *μ*M U0126 for 1 h before stimulation with 10 ng/ml of FGF7 (A) or FGF10 (B). The proliferation of AM-1 cells stimulated with FGF7 or FGF10 was significantly inhibited by adding U0126. Results of the proliferation assay are expressed as mean ± SE. ^*^p<0.05, ^**^p<0.01.

**Figure 6.** Effects of FGF7 and FGF10 neutralizing antibodies on the growth of AM-1 cells and the phosphorylation of p44/42 MAPK. Adding FGF7 or FGF10 neutralizing antibody did not inhibit the proliferation of AM-1 cells (A). The activation of phospho-p44/42 MAPK was not investigated (B). NS, not significant; NA, neutralizing antibody.

**Table I.** Primer sequences for RT-PCR.

Genes	Forward	Reverse
*FGF7*	GCTTGCAATGACATGACTCC	TGCCATAGGAGAAAAGTGGG
*FGF10*	TGTCACCTGCCAAGCCCTT	TACGGGCAGTTCTCCTTCTT
*β-actin*	CATCCTGACCCTCAAGTACCC	GTGGTGGTGAAGCTGTAGCC

**Table II.** Primary antibodies for immunohistochemistry and western blotting.

Antibody (host, clonality, Company)	Purpose	Dilution
FGFR1 (rabbit, polyclonal, Santa Cruz Biotechnology, CA)	IHC	1:150
FGFR2 (rabbit, polyclonal, Santa Cruz Biotechnology, CA)	IHC	1:150
FGF7 (rabbit, polyclonal, Santa Cruz Biotechnology, CA)	IHC	1:150
FGF7 (rabbit, polyclonal, Abcam, Cambridge, UK)	WB	1:200
FGF10 (rabbit, polyclonal, Santa Cruz Biotechnology, CA)	IHC	1:150
FGF10 (goat, polyclonal, Peprotech Inc., Rocky Hill, NJ)	WB	1:200
p-p44/42 MAPK (Thr202/Tyr204) (rabbit, polyclonal, Cell Signaling, Beverly, MA)	WB	1:1,000
Akt (rabbit, polyclonal, Cell Signaling, Beverly, MA)	WB	1:1,000
p-Akt (Ser473) (rabbit, polyclonal, Cell Signaling, Beverly, MA)	WB	1:1,000
Actin (mouse, monoclonal, Amersham, Buckinghamshire, UK)		

IHC, immunohistochemistry; WB, western blotting.

**Table III.** Results of immunohistochemical staining in the ameloblastoma specimens.

Immunoreactivity	FGF7			FGF10			FGFR1			FGFR2		
			
	−	+	++	−	+	++	−	+	++	−	+	++
Follicular type (n=18)												
Tumor cells	0 (0)	16 (88.9)	2 (11.1)	0 (0)	14 (77.8)	4 (22.2)	0 (0)	2 (11.1)	16 (88.9)	0 (0)	0 (0)	18 (100)
Stromal cells	0 (0)	0 (0)	18 (100)	0 (0)	0 (0)	18 (100)	0 (0)	0 (0)	18 (100)	18 (100)	0 (0)	0 (0)
Plexiform type (n=8)												
Tumor cells	0 (0)	6 (75.0)	2 (25.0)	0 (0)	6 (75.0)	2 (25.0)	0 (0)	2 (25.0)	6 (75.0)	0 (0)	0 (0)	8 (100)
Stromal cells	0 (0)	0(0)	8 (100)	0 (0)	0 (0)	8 (100)	0 (0)	4 (50.0)	4 (50.0)	8 (100)	0 (0)	0 (0)
Basal cell type (n=4)												
Tumor cells	0 (0)	2 (50.0)	2 (50.0)	0 (0)	2 (50.0)	2 (50.0)	0 (0)	1 (25.0)	3 (75.0)	0 (0)	0 (0)	4 (100)
Stromal cells	0 (0)	0 (0)	4 (100)	0 (0)	0 (0)	4 (100)	0 (0)	0 (0)	4 (100)	4 (100)	0 (0)	0 (0)
Desmoplastic type (n=2)												
Tumor cells	2 (100)	0 (0)	0 (0)	2 (100)	0 (0)	0 (0)	0 (0)	2 (100)	0 (0)	0 (0)	2 (100)	0 (0)
Stromal cells	0 (0)	2 (100)	0 (0)	0 (0)	2 (100)	0 (0)	0 (0)	2 (100)	0 (0)	0 (0)	2 (100)	0 (0)

Immunohistochemical reactivity: (−), negative; (+), weakly positive; (++), strongly positive.
